The article "The X Files: “The Mystery of X Chromosome Instability in Alzheimer’s Disease”" was published in 2020. Journal: Front Genet.

# The X Files: “The Mystery of X Chromosome Instability in Alzheimer’s Disease”

**DOI:** 10.3389/fgene.2019.01368

**Published:** 2020-01-28

**Authors:** Vladan P. Bajic, Magbubah Essack, Lada Zivkovic, Alan Stewart, Sonja Zafirovic, Vladimir B. Bajic, Takashi Gojobori, Esma Isenovic, Biljana Spremo-Potparevic

**Affiliations:** ^1^Laboratory for Radiobiology and Molecular Genetics, Vinca Institute of Nuclear Sciences, University of Belgrade, Belgrade, Serbia; ^2^Computational Bioscience Research Center (CBRC), Computer, Electrical and Mathematical Sciences and Engineering (CEMSE) Division, King Abdullah University of Science and Technology (KAUST), Thuwal, Saudi Arabia; ^3^Department of Physiology, Faculty of Pharmacy, University of Belgrade, Belgrade, Serbia; ^4^School of Medicine, University of St Andrews, St Andrews, United Kingdom; ^5^Biological and Environmental Sciences and Engineering Division (BESE), King Abdullah University of Science and Technology (KAUST), Thuwal, Saudi Arabia

**Keywords:** X chromosome, Alzheimer’s disease, sex chromosome dosage, protocadherin 11, centromere instability

## Abstract

Alzheimer’s disease (AD) is a neurodegenerative disease that affects millions of individuals worldwide and can occur relatively early or later in life. It is well known that genetic components, such as the amyloid precursor protein gene on chromosome 21, are fundamental in early-onset AD (EOAD). To date, however, only the apolipoprotein E4 (ApoE4) gene has been proved to be a genetic risk factor for late-onset AD (LOAD). In recent years, despite the hypothesis that many additional unidentified genes are likely to play a role in AD development, it is surprising that additional gene polymorphisms associated with LOAD have failed to come to light. In this review, we examine the role of X chromosome epigenetics and, based upon GWAS studies, the PCDHX11 gene. Furthermore, we explore other genetic risk factors of AD that involve X-chromosome epigenetics.

## Introduction

In the first two decades of the 21st century, the proportion of individuals living with Alzheimer’s disease (AD) [AD (MIM: 104300)] has been on the rise with an increasingly aging population. Today, two basic forms of AD exist, early-onset AD (EOAD) and late-onset AD (LOAD). EOAD correlates with the occurrence of mutations on specific genes that have given rise to inherited forms of the disease, whilst LOAD - which occurs later in life - has no specified etiology (Smith, 1998; Selkoe, 2001). Familial studies have identified a point mutation associated with EOAD on chromosome 21. This mutation is located in a gene called amyloid precursor protein (APP), and all members of these families show signs of the Alzheimer’s phenotype at a relatively early stage of life (Wiseman et al., 2018). Novel mutations located on chromosomes 14 and 1 in genes encoding presenilin-1 and presenilin-2 have also been identified in EOAD (Guven et al., 2019). Unfortunately, specific genetic determinants that can explain the high prevalence of LOAD have yet to be identified.

The article "The X Files: “The Mystery of X Chromosome Instability in Alzheimer’s Disease”" was published in 2020. Journal: Front Genet.

Today we are aware that EOAD comprises only 1-3% of all AD cases (Smith, 1998; Selkoe, 2001; Bekris et al., 2010). In LOAD subjects, disease prevalence changes with age; 5% after 65 years of age, 20% after 75 years of age, 30% after 80 years of age (Bekris et al., 2010). Also women are twice as likely to suffer from AD than men (Pike, 2017). This prevalence is suggested to be due to differences in the life expectancy between males and females and to hormonal status (Vest and Pike, 2013; Pike, 2017). Studies with twins clearly signal that a strong genetic component is present in LOAD cases (Gatz et al., 2006; Seripa et al., 2009). Various genes have been implicated in AD and identified by using genetic approaches, such as Genome-Wide Association Studies (GWAS). However, the only “single gene” risk factor for LOAD without opposition in the research community concerns the gene encoding apolipoprotein E4 (Giri et al., 2017). In LOAD, the percentage of individuals carrying the at-risk allele of the ApoE4 gene was found to be between 20% and 70%, suggesting that there are additional genetic, and perhaps also epigenetic, factors that underlie the development of LOAD (Slooter et al., 1998; Giri et al., 2017). Carrasquillo et al. (Carrasquillo et al., 2009) found that an alteration of a single-nucleotide polymorphism (SNP; rs5984894) on the Xq21.3 in a gene called protocadherin 11 (PCDH11X) in a cohort of women, was significantly associated with LOAD (**Figure 1**). Other GWAS, however, have been unable to confirm the existence of these connections (Beecham et al., 2010; Wu et al., 2010; Miar et al., 2011; Chung et al., 2013). We hypothesize that one of the possible answers to these observed genetic discrepancies is based on the epigenetics of the X chromosome.

**Figure 1:** The genetic position of the PCDH11X on the X chromosome.

We have previously identified centromere impairment or premature centromere separation (PCS) of the X chromosome in neuronal nuclei of the cerebral cortex in AD women (Spremo-Potparevic et al., 2008). In addition, Yurov et al. discovered X chromosome aneuploidy in AD-affected neurons (Yurov et al., 2014), which suggests that premature centromere separation is a mechanism of X chromosome instability (Spremo-Potparevic et al., 2008). Epigenetically, chromosome X can be affected by skewed X chromosome inactivation, asynchronous replication patterns of the inactive X chromosome (Xi), X-inactivation escape, aneuploidy, and premature centromere separation. All these epigenetic X chromosome changes could potentially affect X chromosome genes through changes in sex chromosome dosage (SCD), and consequently promote AD pathogenesis (Amiel et al., 1998; Gribnau et al., 2005; Ahn and Lee, 2008; Spremo-Potparevic et al., 2008; Hong and Reiss, 2014; Mugford et al., 2014; Yurov et al., 2014; Bajic et al., 2015a; Balaton and Brown, 2016; Le Gall et al., 2017; Graham et al., 2019). Raznahan et al. found recently that sex chromosome dosage not only influenced the adjacent sex chromosomes X and Y, but also autosomal gene expression (Raznahan et al., 2018).

The article "The X Files: “The Mystery of X Chromosome Instability in Alzheimer’s Disease”" was published in 2020. Journal: Front Genet.

### The X Chromosome Is Unique

In women, there is a systematic demand to compensate for SCD by silencing one of the copies of the X chromosome. With two X-chromosomes, women are more prone to inheriting potentially deleterious mutations in X-encoded genes, which, because of Xi, may all be expressed in different cells. The first finding of inactivation of the X chromosome was reported by Lyon, (1961). It was found that one of the X chromosomes, paternal or maternal, was always inactivated, suggesting that an inactivation mechanism only allows active transcription at one X chromosome (Splinter et al., 2011). This process of X-chromosome inactivation (XCI) evolved as a mechanism to regulate gene dosage. As a compensation mechanism, it does not affect all genes equally, and those genes that are not affected are known to escape XCI [termed escapees; (Pessia et al., 2012)].

Human embryos initially have non-random imprinted XCI, where the X-chromosome from the mother remains active, and XCI applies only to the X-chromosome inherited from the father. The imprint is not constant; XCI resets at the embryonic implantation stage. At this point the XCI reset leaves the maternal and paternal X open to random inactivation (Sun and Lee, 2006). Because XCI at this stage is random it causes most women to be mosaic for two cell lines, one harboring the active chromosome, the paternal X, and the other the maternal X. The randomness of this process causes an XCI ratio of approximately 50%:50% to be associated with the two cell lines in the female population. However, on rare occasions, in approximately 9% of the female population, a bias towards one of the two X chromosomes produces a skewed ratio (> 80%:20%; (Amos-Landgraf et al., 2006). In this regard, Renault et al., analyzed the distribution of X-inactivation patterns (the relative abundance of the two cell populations) in a large cohort study of normal females, and reported that human XCI distribution pattern is more genetically influenced in comparison to the Xi model, which suggests a completely random selection of XCI (Renault et al., 2013).

The article "The X Files: “The Mystery of X Chromosome Instability in Alzheimer’s Disease”" was published in 2020. Journal: Front Genet.

The genetically influenced selection of XCI may be indicative of mutations in genes (Orstavik, 2009; Shvetsova et al., 2019), suggesting the inactive X chromosome often harbors the mutated allele of an X-linked gene. This would mean that with a 50%:50% XCI ratio, wild type cells generally ameliorate disease phenotypes. Changes in the XCI ratio towards an increased expression of mutated genes can increase disease phenotype severity, as it is in the case of female hemophilia A (Renault et al., 2007), and sideroblastic anemia (Cazzola et al., 2000), where the majority of cells express the mutated allele. Changes in the XCI ratio where expression of the mutated allele is increased to exhibit the disease phenotype can also occur, as in Rett syndrome. In this case, the hemizygous mutation of the methyl-CpG–binding protein 2 (MeCP2) gene in males causes lethality, while the MeCP2 heterozygous mutation in females weakens such phenotypic consequences. It seems that the loss of MeCP2 function contributes to Rett syndrome, while the gain in MeCP2 dosage does not necessarily ameliorate the disease phenotype but may manifest as a less aggressive form in other neurological diseases. Increased expression of MeCP2 was found to be associated with other neurological diseases, such as AD and Huntington’s disease (Amir et al., 1999; Ausio et al., 2014; McFarland et al., 2014; Maphis et al., 2017).

Xi acquires several features of heterochromatin, such as hypermethylation, hypercondensation, altered replication patterns (late *vs.* early), and depletion of acetylated histones (Chow and Brown, 2003; Ng et al., 2007). Methylation patterns have been extensively used to determine the inactive chromosome (Shvetsova et al., 2019), enabling an analysis of non-random inactivation processes in diseases that are X chromosome-linked (Yuan et al., 2015). In our published study we suggest that changes in the inactivation patterns of the X-chromosome could have an impact on AD pathogenesis (Bajic et al., 2015a).

## Brain and the X Chromosome

The X chromosome harbors 3-5% of all the genes in a genome (Skuse, 2005). There has been a debate on how many genes reside on the X chromosome and how many genes are expressed in the brain alone, compared to genes that are X-linked and expressed in the placenta, testes, muscles, and ovary. It is estimated that between 1,100 and 1,500 genes are present on the X chromosome (Skuse, 2005; Laumonnier et al., 2007). By using the Mart View software it was found that 1,500 X-linked genes are expressed in the brain, which represent numerous candidate genes that could be responsible for X-linked brain diseases (Laumonnier et al., 2007). Many of the proteins expressed from the genes linked to the X chromosome represent channels, receptors, repair, transcription factors, and DNA/RNA binding proteins. Most of these proteins are located in the postsynaptic cleft and postsynaptic density (PSD) and are regulated through signaling complexes (Nguyen and Disteche, 2006; Laumonnier et al., 2007). It is intriguing that even if the X chromosome harbors 3-5% of all the genes, it is responsible for 10% of all diseases with Mendelian inheritance (Germain, 2006).

The article "The X Files: “The Mystery of X Chromosome Instability in Alzheimer’s Disease”" was published in 2020. Journal: Front Genet.

Another aspect that makes the X chromosome unique is that it harbors a higher proportion of brain-expressed miRNAs than would be expected (Goncalves et al., 2019), with 20% of these related to autoimmune diseases such as rheumatoid arthritis and systemic lupus erythematosus (Khalifa et al., 2016). Most of these miRNA are clustered, for example, miR532/188, miR-221/222, miR-98/Let7f, and miR-363/106a/20b/92a (DeMarco et al., 2019; Goncalves et al., 2019). Many of these are also intronic and it is believed that they are co-transcribed and co-expressed with other genes linked to chromosome X (deleted X-linked genes) and may be susceptible to SCD, skewing, and Xi escape processes. It is important to point out that inflammation and altered immunity are features of AD (Forloni et al., 1992; Hauss-Wegrzyniak et al., 1998; Eikelenboom et al., 2000; McGeer and McGeer, 2002; Castellani et al., 2008; Krstic et al., 2012; Bajic et al., 2015c; Regen et al., 2017).

How these X-linked genes interact with genes controlling the immune system in AD is still unknown. For individual genes involved in diseases of the brain, a more complex hypothesis is that interplay occurs in disease genes embedded in multiprotein neuronal complexes. Many of the most important components of neuronal complexes are encoded on the X chromosome (Laumonnier et al., 2007). Such complexes, which are essential for neuronal plasticity, cognitive processes, and cell signaling, are thought to be in the PSD cleft (Muddashetty et al., 2011; Yudowski et al., 2013). Taking N-methyl-D-aspartate receptor/membrane-associated guanylate kinase-associated signaling complex/(NRC/MASC) as an example; combining its 185 proteins and with the other proteins in PSD gives a total of 1100 proteins. The X chromosome plays an essential role, and the percentage of genes related to synaptic plasticity, some 86% of all the genes in NRC/MASC are genes linked to chromosome X (Grant et al., 2005; Laumonnier et al., 2007). It is interesting that these genes are also presented or expressed in human cognitive disorders (Grant et al., 2005; Pocklington et al., 2006; Fernandez et al., 2009; Tam et al., 2009). An analysis of the number of altered proteins in X-linked mental retardation disorders shows that from 69 genes currently known, 19 (or 28%) of these genes belong to postsynaptic proteins (Laumonnier et al., 2007). The same pattern is conserved in the mouse X chromosome, and this suggests a network of multiprotein complexes functioning as integrated entities or complex molecular machines. If one component of this complex machinery is disrupted, the whole complex/network fails thus impairing the overall role of the multiprotein complex in processes of cognition (Grant et al., 2005; Nguyen and Disteche, 2006; Pocklington et al., 2006; Laumonnier et al., 2007; Fernandez et al., 2009; Tam et al., 2009).

The article "The X Files: “The Mystery of X Chromosome Instability in Alzheimer’s Disease”" was published in 2020. Journal: Front Genet.

### X-Linked miRNA and the Brain

The X chromosome is enriched in ncRNAs and harbors several miRNAs essential to brain function (Goncalves et al., 2019). It is important to note that miRNAs not only affect mRNA through translation repression but also work through other ncRNAs, such as lncRNAs and circRNAs, affecting downstream genes (Khalifa et al., 2016; DeMarco et al., 2019; Goncalves et al., 2019). Bian et al. revealed that a miRNA located on the X chromosome, a miR-374 family member, plays a role in cell growth and differentiation not only in various cancers, but also in AD. This miR-374 member is located at the X chromosome inactivation center and targets the VEGF, PTEN, Wnt, and Fas signaling pathways (Bian et al., 2019). Importantly, the PTEN pathway is of importance to the progression of AD through a mechanism that includes altered autophagy (Wani et al., 2019), mitophagy (Fang et al., 2019), and apoptosis (Cui et al., 2017). A report by Manzine et al. suggested that miR-374 directly targets the beta-secretase 1 to regulate the progress of AD, as the levels of miR-374 were significantly decreased in comparison to controls (Manzine et al., 2018). In addition to miR-374, several miRNAs have also been found to correlate to X chromosome-linked intellectual disability syndrome, and among them are miR-223-3p, miR-362-5p, miR-504-5p.1, miR-361-5p, miR-505-3p.1 and miR-505-3p.2. All these miRNAs act as key regulators of genes linked to chromosome X but also of many autosomal intellectual disability genes that are connected in a complex network (Goncalves et al., 2019).

In the future, it is hoped that further work will reveal the extent to which genes on the X chromosome and miRNAs expressed in the brain, that together regulate processes including nervous system development, cell proliferation and transcription regulation, are altered by X chromosome skewing and asynchronous replication, which lead to aneuploidy and deregulation of cohesion dynamics in AD. Also, RNA genes that are linked to the X chromosome are prone to escape inactivation of the X chromosome (Peeters et al., 2019). These epigenetic processes may prove to be gender-associated as research shows that expression of an X-linked miRNA in rheumatoid arthritis is more prevalent in women than in men (Khalifa et al., 2016).

The article "The X Files: “The Mystery of X Chromosome Instability in Alzheimer’s Disease”" was published in 2020. Journal: Front Genet.

## PCDH11X

Carrasquillo et al. previously identified an SNP (rs 5984894) on the X chromosome (Xq21,3) in a gene called PCDH11X (Carrasquillo et al., 2009). This locus is associated with LOAD in women of European origin from the USA. The PCDH11X gene encodes the protein, protocadherin 11. Women who are homozygous for this SNP have a greater risk of developing AD, not only when compared to women without the SNP, but also when compared to women that are heterozygotes, and male hemizygotes (Carrasquillo et al., 2009). Zubenko et al. reported that the DXS1047 genotype is correlated with AD (Zubenko et al., 1999) and that this genotype is associated with the PCDH11X gene (Zubenko et al., 1998). The results from the same authors indicate an association between the variation in the PCDH11X gene and the risk of acquiring AD, but these results have not been confirmed in other GWAS (Beecham et al., 2010; Wu et al., 2010; Miar et al., 2011). Our suggestion is that these discrepancies in GWAS results may well be due to the changes in the epigenetics of the X chromosome.

### Does PCDH11X Escape X Inactivation?

Pseudoautosomal genes and functional Y chromosome orthologues (X-linked genes with Y homology) tend to escape X inactivation (Disteche et al., 2002; Brown and Greally, 2003). Sudbrak et al. reported that PCDH11X expression might also escape X inactivation, and this assumption was verified by using an X chromosome-specific cDNA microarray where elevated expression of PCDH11X was identified in cells expressing multiple X chromosomes (Sudbrak et al., 2001). Lopes et al. indirectly found that PCDH11X expression was higher in women than in men by looking at CpG islands and their methylation patterns. By using bisulfite sequencing analysis, the same authors found the absence of CpG island methylation on both the active and the Xi chromosomes and that these processes coincide with possible PCDH11X escape from X inactivation (Lopes et al., 2006). Another study found that PCDH11X can undergo asynchronous replication, and that PCDHX11 is also prone to escape the inactivation process (Wilson et al., 2007). Replication asynchrony of the X pseudoautosomal locus has been identified (Vorsanova et al., 2001), and suggests that other genes that replicate asynchronously are also prone to escape inactivation (Anderson and Brown, 2005; Carrel and Willard, 2005; Escamilla-Del-Arenal et al., 2011).

The article "The X Files: “The Mystery of X Chromosome Instability in Alzheimer’s Disease”" was published in 2020. Journal: Front Genet.

### PCDH11X Asynchronous Replication

Xi is associated with a sequence of epigenetic modifications (Chow and Brown, 2003), and goes through a phase of changes involving DNA methylation and histone modification resulting in Xi condensation in a body called the Barr body. This results in changes in DNA replication – more specifically, the Xi in the S phase replicates later than its active counterpart. Imperfect chromosome replication can be a consequence of “escapees” (genes that escape the inactivation process). Such genes include hypoxanthine-guanine phosphoribosyltransferase and Fragile X-chromosome genes that display asynchronicity. The X-inactive-specific transcript (Xist) gene (important for inactivation) that is expressed from the Xi also replicates asynchronously (Boggs and Chinault, 1994; Aladjem and Fu, 2014). Wilson et al. reported that PCDH11X displays replication asynchrony in both female and male cells (Wilson et al., 2007). The data from these authors, together with those from others (Orstavik, 2009), show that a complex relationship exists between X-inactivation, replication asynchrony, and the status of expression of individual genes on chromosome X (Bajic et al., 2008; Bajic et al., 2009).

It thus appears that synchronous replication occurs more frequently than previously thought, and is found not only through imprinting, but also through randomized monoallelic expression, pathologies, and tandem duplications (Wilson et al., 2007). Clinically, an increase in asynchronous replication increases the risk in women for aneuploidy (Amiel et al., 2000). The relationship between centromere instability, control of replication, and nondisjunction are best exemplified by the fact that young women that have children with Down’s syndrome have twice the risk of developing AD (Hardy et al., 1989; Goate et al., 1990; Fidani et al., 1992; Schellenberg et al., 1992; Schupf et al., 1994; Petersen et al., 2000; Schupf et al., 2001; Migliore et al., 2006; Migliore et al., 2009; Iourov et al., 2010; Goate and Hardy, 2012).

Chromosomes 21, X, and 18 were primarily affected, showing repeated non-disjunction and centromere impairment (Potter and Geller, 1996; Geller and Potter, 1999; Petersen et al., 2000; Migliore et al., 2006; Migliore et al., 2009; Iourov et al., 2010; Potter, 2016). We suggest that X chromosome replication asynchrony is likely to lead to accelerated instability of chromosome X in AD (Bajic et al., 2009).

## Sex Chromosome Dosage (SCD): an Engine of Stability

The crosstalk that exists between X chromosomes and autologous genes is a relatively new paradigm that has emerged as a result of the biology of sex differences, and gives rise to the question of how SCD shapes the genome function. To explore this, human sex aneuploidies were analyzed from a genome-wide expression dataset by Raznahan et al. where they found a dosage sensitivity of the X-Y chromosome pair resulting in increased expression of genes that decrease X/Y chromosomal dosage (Raznahan et al., 2018). The most interesting finding was that X-linked genes were found to regulate co-expression of networks of autosomal genes that are SCD-sensitive and, in addition to these findings, suggest that the autosomal genes and their corresponding networks are crucial for cellular functions. This highlights the potential of SCD to affect the occurrence of disease.

The article "The X Files: “The Mystery of X Chromosome Instability in Alzheimer’s Disease”" was published in 2020. Journal: Front Genet.

The most common aneuploidy in AD is XO mosaicism (Spremo-Potparevic et al., 2004; Spremo-Potparevic et al., 2008; Yurov et al., 2014; Spremo-Potparevic et al., 2015). In respect to SCD and the XO status, Raznahan et al. have demonstrated up-regulation of the protein networks, noncoding RNA metabolism, suppression of the cell cycle, changes in regulation of DNA/chromatin organization, glycolysis, and response to stress (Raznahan et al., 2018). Changes in these collective networks through XO and supernumerary XXY, and XXYY syndromes may enhance the risk of AD (Raznahan et al., 2018; Graham et al., 2019).

There is a small but constant number of neuronal cells that express a different number of chromosomes, such as aneuploidy (Iourov et al., 2006; Yurov et al., 2007; Iourov et al., 2008; Iourov et al., 2009; Yurov et al., 2014), but also copy number variation on chromosome 21, which is crucial in AD (Cai et al., 2014), DNA content variation (Madrigal et al., 2007; Westra et al., 2010), and LINE elements (Evrony et al., 2012).

Mosaic aneuploidy in the brain revealed that not only was chromosome 21 affected in AD, but also that the X chromosome was found to be supernumerary and presumed to be affected through a mechanism that involves altered cohesion/cohesin dynamics (Spremo-Potparevic et al., 2004; Spremo-Potparevic et al., 2008; Bajic et al., 2009; Zivković et al., 2010; Zivkovic et al., 2013; Yurov et al., 2014; Bajic et al., 2015b; Spremo-Potparevic et al., 2015; Yurov et al., 2019).

Yurov et al. (2014) suggested that chromosome 21 might not be the only chromosome to influence changes in genome stability of a neuron, which leads to a cascade of processes that result in neuronal loss. The finding that affected brains show a two-fold increase in X chromosome aneuploidy in the hippocampus and cerebrum - areas of the brain most affected by AD - suggesting that altered sex chromosome dosage plays a role in the large scale genomic variation in neuronal cells in AD compared to controls. These results have been recently corroborated by the finding that the sex chromosomes were distinct from autosomes in the dorsolateral prefrontal cortex and that X chromosome aneuploidy was associated with a faster rate of cognitive decline which is a hallmark of AD (Graham et al., 2019). Therefore, X chromosome aneuploidy may contribute to aging, but also to processes leading to pathological changes in brains affected by AD.

The article "The X Files: “The Mystery of X Chromosome Instability in Alzheimer’s Disease”" was published in 2020. Journal: Front Genet.

Previously we proposed the “post-mitotic state-maintained protein hypothesis” where we distinguished aneuploization in the brain as constitutional aneuploidy with non-pathological diversification of the neurons (Bajic et al., 2015b). These aneuploidogenic processes are balanced with cohesin and cohesion-related proteins. Alteration of this balance develops as a link between neuronal development and chromosomal instability, intracellular diversity and human brain diseases including AD (Hong and Reiss, 2014). Looking closely at the overall somatic mosaicism found in the brain, we, together with others, suggest that micro aneuploidy or segmental aneuploidy is a more proper measure of changes in gene dosage leading to AD (Dierssen et al., 2009). These processes are heavily realized when looking at SCD effects on gene expression in humans (Raznahan et al., 2018).

An additional complexity of genome mosaicism in the brain relates to findings concerning DNA and gene copy number variations. Regional variations of DNA content has been identified with higher DNA content found in the frontal cortex and cerebellum compared with other brain regions (Westra et al., 2010). Copy number variations may be considered as an independent genetic factor not related to other genomic changes, suggesting its plays a role in neurodevelopmental disorders in patients with sex chromosome aneuploidies (Haack et al., 2013; Le Gall et al., 2017). It has been reported that 11% of neurons in the brain cortex exhibit a DNA content that is above the diploid level (Fischer et al., 2012), and similar findings have also been reported in the AD brain (Ueberham and Arendt, 2005; Arendt et al., 2010; Yurov, 2017; Barrio-Alonso et al., 2018). These somatic gene variations in neurons appear to be generated by chromosome segregation defects. Some of these cells are expelled by apoptosis, but several cells are introduced as a pool of variability of the neuronal genome. These cell populations are thus vulnerable in the sense that they are more prone to genome instability and thus may contribute to age-related mental disorders, such as AD. Gómez-Ramos et al. presented distinct X-chromosome single nucleotide variants from some sporadic AD samples (Gómez-Ramos et al., 2015). In samples from LOAD patients, a higher number of single nucleotide variants in genes present at the X chromosome were identified using exome sequencing compared to age-matched controls. Two genes that were not previously described as risk factors, UBE2NL and ATXN3L, were found to have variants important for the ubiquitin pathway in LOAD (Gómez-Ramos et al., 2015).

The article "The X Files: “The Mystery of X Chromosome Instability in Alzheimer’s Disease”" was published in 2020. Journal: Front Genet.

Maintenance of the interphase state in neurons is an active process. The 3D organization of the genome is correlated to gene expression in the interphase. In the 3D domain, chromosomes occupy preferential positions by self-organizing into topologically-associated domains, which may change due to the cell lineage or stage of the organism (Laskowski et al., 2019). There is a possible exchange between the inactive and active chromosome in gene regulatory information. Cohesin is indirectly associated with the Xi 3D position in the genome. Minajigil et al. reported that a reaction between Xist and cohesins results in the repulsion of the latter from Xi, thus changing its 3D shape (Minajigi et al., 2015). The Xi is much more complex, and it also represents a reservoir of genes that could replace mutated genes from the active X chromosome. At present, this untapped potential known as the X interactome requires further investigation (Minajigi et al., 2015). Progress in understanding the Xist interactome requires more understanding of how it is used and how epigenetically-regulated long ncRNAs potentially influence disease. By utilizing a specific technique named iDRiP, some 200 proteins in the Xist interactome were identified (Minajigi et al., 2015). Most of the proteins are from several categories, such as cohesins, condesins, topoisomerases, RNA helicase, histone modifiers, methyltransferases, nuclear matrix proteins, and nucleoskeletal factors. Cohesin may play a more important role in the complex relationship between the Xi and active X chromosome (Minajigi et al., 2015). Even though these processes are an important mechanism of diversity, alterations may lead to an increased structural and topological variation of the genome in the brain, enhancing the susceptibility of affected neurons to genome instability that may lead to AD (Bajic et al., 2015b; Graham et al., 2019; Yurov et al., 2019).

A number of publications have reported mislocalization of some critical proteins responsible for chromatin organization and epigenetic modifications in brain diseases including AD (Gill et al., 2007; Lu et al., 2014; Luperchio et al., 2014; Quinodoz and Guttman, 2014; Guo et al., 2015; Mastroeni et al., 2015; Pombo and Dillon, 2015; Sen et al., 2015; Winick-Ng and Rylett, 2018).

The article "The X Files: “The Mystery of X Chromosome Instability in Alzheimer’s Disease”" was published in 2020. Journal: Front Genet.

All these data suggest, that in AD chromatin, organizers are deregulated and chromatin topology is changed in a manner that alters gene expression leading to synaptic dysfunction, a major pathological change in AD, and consequently neurodegeneration (Gill et al., 2007; Lu et al., 2014; Luperchio et al., 2014; Quinodoz and Guttman, 2014; Guo et al., 2015; Mastroeni et al., 2015; Pombo and Dillon, 2015; Sen et al., 2015; Winick-Ng and Rylett, 2018).

Xist RNA can act as a scaffold for proteins required to maintain the inactive state of neurons. It has been shown that it can act as a repulsion mechanism that expels architectural factors such as cohesins in order to avoid unwanted chromatin conformation that could increase unfavorable transcription (Raznahan et al., 2018). Minajigi et al. suggest that Xi RNA plays an important role in the organization of how chromosomes are regulated into chromosome territories and that Xi inactivation is fundamentally important in these processes (Minajigi et al., 2015). It could be suggested that X chromosome instability found in AD may result in changes in the Xi pattern, Xi escapees, SCD, and consequently changes in the topological organization, thus altering chromatin organization that may affect already other genes related to AD (**Figure 2**).

**Figure 2:** X chromosome instability, Sex Chromosome Dosage, Topological changes of Chromosomes, and its possible role in AD.

The cohesin-associated protein, shugoshin-1, seems to be fundamental in repressing the accumulation of amyloid-β and Tau phosphorylation in shugoshin-1 gene (Sgo1) haploinsufficient mice (Rao et al., 2018).

## Summary

Conflicting results from studies of the PCDH11X gene in AD could be explained by cohort size, ethnicity, and environmental factors *per se* but also by the influence of X chromosome epigenetics. Thus, GWAS of sex chromosomes should take into account any alterations of the epigenetic processes in the X chromosome (Schurz et al., 2019).

The findings that chromosome X expresses all of the somatic genomic neuronal variability properties and can *de novo* express several epigenetic mechanisms suggest that the X chromosome instability phenotype may be viewed as an important risk factor in AD pathogenesis.

## Author Contributions

All authors (VPB, ME, LZ, AS, SZ, VBB, TG, EI, and BS-P) contributed to the design and writing of the manuscript. VPB and SZ designed the figures.

## Funding

This work is part of the collaboration between the Laboratory of Radiobiology and Molecular Genetics, Vinca Institute of Nuclear Sciences, University of Belgrade, Belgrade, Serbia and King Abdullah University of Science and Technology (KAUST), Computational Bioscience Research Center (CBRC), Thuwal, Saudi Arabia. This work has been supported by grants No. 173033 (EI) and No. 173034 (VPB) from the Ministry of Education, Science and Technological Development, Republic of Serbia and by the KAUST grant OSR#4129 (to EI and VBB), which also supported SZ and VPB. VBB has been supported by the KAUST Base Research Fund (BAS/1/1606-01-01), while VBB and ME have been supported by KAUST Office of Sponsored Research (OSR) grant no. FCC/1/1976-17-01. TG has been supported by the King Abdullah University of Science and Technology (KAUST) Base Research Fund (BAS/1/1059-01-01).

The article "The X Files: “The Mystery of X Chromosome Instability in Alzheimer’s Disease”" was published in 2020. Journal: Front Genet.

## Conflict of Interest

The authors declare that the research was conducted in the absence of any commercial or financial relationships that could be construed as a potential conflict of interest.

## Abbreviations

AD, Alzheimer’s disease; EOAD, Early onset AD; GWAS, genome-wide association studies; LOAD, Late onset AD; NRC/MASC, N-methyl-D-aspartate receptor complex/membrane-associated guanylate kinase-associated signaling complex; PCDH11X, protocadherin 11; PSD, postsynaptic density; SCD, Sex Chromosome Dosage; Xist, X-inactive-specific transcript gene; Xi, inactive X chromosome.

## References

[B1] AhnJ.LeeJ. (2008). X chromosome: X inactivation. Nature Education 1, 24.

[B2] AladjemM. I.FuH. (2014). A new light on DNA replication from the inactive X chromosome. Bioessays 36, 591–597. 10.1002/bies.201400021 24706495PMC4153745

[B3] AmielA.AviviL.GaberE.FejginM. D. (1998). Asynchronous replication of allelic loci in down syndrome. Eur. J. Hum. Genet. 6, 359–364. 10.1038/sj.ejhg.5200199 9781044

[B4] AmielA.ReishO.GaberE.KedarI.DiukmanR.FejginM. (2000). Replication asynchrony increases in women at risk for aneuploid offspring. Chromosome Res. 8, 141–150. 10.1023/a:1009246603868 10780703

[B5] AmirR. E.Van den VeyverI. B.WanM.TranC. Q.FranckeU.ZoghbiH. Y. (1999). Rett syndrome is caused by mutations in X-linked MECP2, encoding methyl-CpG-binding protein 2. Nat. Genet. 23, 185–188. 10.1038/13810 10508514

[B6] Amos-LandgrafJ. M.CottleA.PlengeR. M.FriezM.SchwartzC. E.LongshoreJ. (2006). X chromosome-inactivation patterns of 1,005 phenotypically unaffected females. Am. J. Hum. Genet. 79, 493–499. 10.1086/507565 16909387PMC1559535

[B7] AndersonC. L.BrownC. J. (2005). Epigenetic predisposition to expression of TIMP1 from the human inactive X chromosome. BMC Genet. 6, 48. 10.1186/1471-2156-6-48 16194278PMC1262707

[B8] ArendtT.BrucknerM. K.MoschB.LoscheA. (2010). Selective cell death of hyperploid neurons in Alzheimer’s disease. Am. J. Pathol. 177, 15–20. 10.2353/ajpath.2010.090955 20472889PMC2893646

The article "The X Files: “The Mystery of X Chromosome Instability in Alzheimer’s Disease”" was published in 2020. Journal: Front Genet.

[B9] AusioJ.Martinez de PazA.EstellerM. (2014). MeCP2: the long trip from a chromatin protein to neurological disorders. Trends Mol. Med. 20, 487–498. 10.1016/j.molmed.2014.03.004 24766768

[B14] BajicV. P.Spremo-PotparevicB.ZivkovicL.DjelicN.SmithM. A. (2008). Is the time dimension of the cell cycle re-entry in AD regulated by centromere cohesion dynamics? Biosci. Hypotheses 1, 156–161. 10.1016/j.bihy.2008.03.006 19122823PMC2612585

[B13] BajicV. P.Spremo-PotparevicB.ZivkovicL.BondaD. J.SiedlakS. L.CasadesusG. (2009). The X-chromosome instability phenotype in Alzheimer’s disease: a clinical sign of accelerating aging? Med. Hypotheses 73, 917–920. 10.1016/j.mehy.2009.06.046 19647374PMC2787990

[B10] BajicV.MandusicV.StefanovaE.BozovicA.DavidovicR.ZivkovicL. (2015a). Skewed X-chromosome inactivation in women affected by Alzheimer’s disease. J. Alzheimers Dis. 43, 1251–1259. 10.3233/JAD-141674 25159673

[B11] BajicV.Spremo-PotparevicB.ZivkovicL.IsenovicE. R.ArendtT. (2015b). Cohesion and the aneuploid phenotype in Alzheimer’s disease: A tale of genome instability. Neurosci. Biobehav. Rev. 55, 365–374. 10.1016/j.neubiorev.2015.05.010 26003528

[B12] BajicV.StanojevicB.ZivkovicL.CabarkapaA.PerryG.ArendtT. (2015c). Cyclin dependent kinase 11, neuroinflammation and alzheimer’s disease: a review. J. Clin. Cell Immunol. 6, 305. 10.4172/2155-9899.1000305

[B15] BalatonB. P.BrownC. J. (2016). Escape Artists of the X Chromosome. Trends Genet. 32, 348–359. 10.1016/j.tig.2016.03.007 27103486

[B16] Barrio-AlonsoE.Hernández-VivancoA.WaltonC. C.PereaG.FradeJ. M. (2018). Cell cycle reentry triggers hyperploidization and synaptic dysfunction followed by delayed cell death in differentiated cortical neurons. Sci. Rep. 8, 14316–14316. 10.1038/s41598-018-32708-4 30254284PMC6156334

[B17] BeechamG. W.NajA. C.GilbertJ. R.HainesJ. L.BuxbaumJ. D.Pericak-VanceM. A. (2010). PCDH11X variation is not associated with late-onset Alzheimer disease susceptibility. Psychiatr. Genet. 20, 321–324. 10.1097/YPG.0b013e32833b635d 20523261PMC2964434

[B18] BekrisL. M.YuC. E.BirdT. D.TsuangD. W. (2010). Genetics of Alzheimer disease. J. Geriatr. Psychiatry Neurol. 23, 213–227. 10.1177/0891988710383571 21045163PMC3044597

[B19] BianH.ZhouY.ZhouD.ZhangY.ShangD.QiJ. (2019). The latest progress on miR-374 and its functional implications in physiological and pathological processes. J. Cell Mol. Med. 23, 3063–3076. 10.1111/jcmm.14219 30772950PMC6484333

[B20] BoggsB. A.ChinaultA. C. (1994). Analysis of replication timing properties of human X-chromosomal loci by fluorescence *in situ* hybridization. Proc. Natl. Acad. Sci. U.S.A. 91, 6083–6087. 10.1073/pnas.91.13.6083 8016119PMC44142

The article "The X Files: “The Mystery of X Chromosome Instability in Alzheimer’s Disease”" was published in 2020. Journal: Front Genet.

[B21] BrownC. J.GreallyJ. M. (2003). A stain upon the silence: genes escaping X inactivation. Trends Genet. 19, 432–438. 10.1016/S0168-9525(03)00177-X 12902161

[B22] CaiX.EvronyG. D.LehmannH. S.ElhosaryP. C.MehtaB. K.PoduriA. (2014). Single-cell, genome-wide sequencing identifies clonal somatic copy-number variation in the human brain. Cell Rep. 8, 1280–1289. 10.1016/j.celrep.2014.07.043 25159146PMC4272008

[B23] CarrasquilloM. M.ZouF.PankratzV. S.WilcoxS. L.MaL.WalkerL. P. (2009). Genetic variation in PCDH11X is associated with susceptibility to late-onset Alzheimer’s disease. Nat. Genet. 41, 192–198. 10.1038/ng.305 19136949PMC2873177

[B24] CarrelL.WillardH. F. (2005). X-inactivation profile reveals extensive variability in X-linked gene expression in females. Nature 434, 400–404. 10.1038/nature03479 15772666

[B25] CastellaniR. J.LeeH. G.ZhuX.PerryG.SmithM. A. (2008). Alzheimer disease pathology as a host response. J. Neuropathol. Exp. Neurol. 67, 523–531. 10.1097/NEN.0b013e318177eaf4 18520771PMC2763411

[B26] CazzolaM.MayA.BergamaschiG.CeraniP.RostiV.BishopD. F. (2000). Familial-skewed X-chromosome inactivation as a predisposing factor for late-onset X-linked sideroblastic anemia in carrier females. Blood 96, 4363–4365. 10.1182/blood.V96.13.4363 11110715

[B27] ChowJ. C.BrownC. J. (2003). Forming facultative heterochromatin: silencing of an X chromosome in mammalian females. Cell Mol. Life Sci. 60, 2586–2603. 10.1007/s00018-003-3121-9 14685685PMC11138508

[B28] ChungS. J.LeeJ. H.KimS. Y.YouS.KimM. J.LeeJ. Y. (2013). Association of GWAS top hits with late-onset Alzheimer disease in Korean population. Alzheimer Dis. Assoc. Disord. 27, 250–257. 10.1097/WAD.0b013e31826d7281 22975751

[B29] CuiW.WangS.WangZ.WangZ.SunC.ZhangY. (2017). Inhibition of PTEN attenuates endoplasmic reticulum stress and apoptosis *via* activation of PI3K/AKT pathway in Alzheimer's disease. Neurochem. Res. 42, 3052–3060. 10.1007/s11064-017-2338-1 28819903

[B30] DeMarcoB.StefanovicS.WilliamsA.MossK. R.AndersonB. R.BassellG. J. (2019). FMRP - G-quadruplex mRNA - miR-125a interactions: implications for miR-125a mediated translation regulation of PSD-95 mRNA. PLoS One 14, e0217275. 10.1371/journal.pone.0217275 31112584PMC6529005

[B31] DierssenM.HeraultY.EstivillX. (2009). Aneuploidy: from a physiological mechanism of variance to Down syndrome. Physiol. Rev. 89, 887–920. 10.1152/physrev.00032.2007 19584316

[B32] DistecheC. M.FilippovaG. N.TsuchiyaK. D. (2002). Escape from X inactivation. Cytogenet. Genome Res. 99, 36–43. 10.1159/000071572 12900543

The article "The X Files: “The Mystery of X Chromosome Instability in Alzheimer’s Disease”" was published in 2020. Journal: Front Genet.

[B33] EikelenboomP.RozemullerA. J.HoozemansJ. J.VeerhuisR.van GoolW. A. (2000). Neuroinflammation and Alzheimer disease: clinical and therapeutic implications. Alzheimer Dis. Assoc. Disord. 14 Suppl 1, S54–S61. 10.1097/00002093-200000001-00009 10850731

[B34] Escamilla-Del-ArenalM.da RochaS. T.HeardE. (2011). Evolutionary diversity and developmental regulation of X-chromosome inactivation. Hum. Genet. 130, 307–327. 10.1007/s00439-011-1029-2 21687993PMC3132430

[B35] EvronyG. D.CaiX.LeeE.HillsL. B.ElhosaryP. C.LehmannH. S. (2012). Single-neuron sequencing analysis of L1 retrotransposition and somatic mutation in the human brain. Cell 151, 483–496. 10.1016/j.cell.2012.09.035 23101622PMC3567441

[B36] FangE. F.HouY.PalikarasK.AdriaanseB. A.KerrJ. S.YangB. (2019). Mitophagy inhibits amyloid-β and tau pathology and reverses cognitive deficits in models of Alzheimer's disease. Nat. Neurosci. 22, 401–412. 10.1038/s41593-018-0332-9 30742114PMC6693625

[B37] FernandezE.CollinsM. O.UrenR. T.KopanitsaM. V.KomiyamaN. H.CroningM. D. (2009). Targeted tandem affinity purification of PSD-95 recovers core postsynaptic complexes and schizophrenia susceptibility proteins. Mol. Syst. Biol. 5, 269. 10.1038/msb.2009.27 19455133PMC2694677

[B38] FidaniL.RookeK.Chartier-HarlinM. C.HughesD.TanziR.MullanM. (1992). Screening for mutations in the open reading frame and promoter of the beta-amyloid precursor protein gene in familial Alzheimer's disease: identification of a further family with APP717 Val–> Ile. Hum. Mol. Genet. 1, 165–168. 10.1093/hmg/1.3.165 1303172

[B39] FischerH. G.MorawskiM.BrucknerM. K.MittagA.TarnokA.ArendtT. (2012). Changes in neuronal DNA content variation in the human brain during aging. Aging Cell 11, 628–633. 10.1111/j.1474-9726.2012.00826.x 22510449

[B40] ForloniG.DemicheliF.GiorgiS.BendottiC.AngerettiN. (1992). Expression of amyloid precursor protein mRNAs in endothelial, neuronal and glial cells: modulation by interleukin-1. Brain Res. Mol. Brain Res. 16, 128–134. 10.1016/0169-328x(92)90202-m 1334190

[B48] Gómez-RamosA.PodlesniyP.SorianoE.AvilaJ. (2015). Distinct X-chromosome SNVs from some sporadic AD samples. Sci. Rep. 5, 18012. 10.1038/srep18012 26648445PMC4673451

[B41] GatzM.ReynoldsC. A.FratiglioniL.JohanssonB.MortimerJ. A.BergS. (2006). Role of genes and environments for explaining Alzheimer disease. Arch. Gen. Psychiatry 63, 168–174. 10.1001/archpsyc.63.2.168 16461860

[B42] GellerL. N.PotterH. (1999). Chromosome missegregation and trisomy 21 mosaicism in Alzheimer's disease. Neurobiol. Dis. 6, 167–179. 10.1006/nbdi.1999.0236 10408806

[B43] GermainD. P. (2006). “General aspects of X-linked diseases,” in Fabry Disease: Perspectives from 5 Years of FOS. Eds. MehtaA.BeckM.Sunder-PlassmannG. (Oxford: Oxford PharmaGenesis). 21290683

The article "The X Files: “The Mystery of X Chromosome Instability in Alzheimer’s Disease”" was published in 2020. Journal: Front Genet.

[B44] GillS. K.IshakM.DobranskyT.HaroutunianV.DavisK. L.RylettR. J. (2007). 82-kDa choline acetyltransferase is in nuclei of cholinergic neurons in human CNS and altered in aging and Alzheimer disease. Neurobiol. Aging 28, 1028–1040. 10.1016/j.neurobiolaging.2006.05.011 16797789

[B45] GiriM.ShahA.UpretiB.RaiJ. C. (2017). Unraveling the genes implicated in Alzheimer's disease. Biomed. Rep. 7, 105–114. 10.3892/br.2017.927 28781776PMC5526178

[B46] GoateA.HardyJ. (2012). Twenty years of Alzheimer's disease-causing mutations. J. Neurochem. 120 Suppl 1, 3–8. 10.1111/j.1471-4159.2011.07575.x 22122678

[B47] GoateA. M.HardyJ. A.OwenM. J.HaynesA.JamesL.FarrallM. (1990). Genetics of Alzheimer's disease. Adv. Neurol. 51, 197–198. 2403711

[B49] GoncalvesT. F.PiergiorgeR. M.Dos SantosJ. M.GusmaoJ.PimentelM. M. G.Santos-ReboucasC. B. (2019). Network profiling of brain-expressed X-chromosomal microRNA genes implicates shared key microRNAs in intellectual disability. J. Mol. Neurosci. 67, 295–304. 10.1007/s12031-018-1235-7 30604382

[B50] GrahamE. J.VermeulenM.VardarajanB.BennettD.De JagerP.PearseR. V., 2nd (2019). Somatic mosaicism of sex chromosomes in the blood and brain. Brain. Res. 1721, 146345. 10.1016/j.brainres.2019.146345 31348909PMC6717667

[B51] GrantS. G. N.MarshallM. C.PageK.-L.CumiskeyM. A.ArmstrongJ. D. (2005). Synapse proteomics of multiprotein complexes: en route from genes to nervous system diseases. Hum. Mol. Genet. 14, R225–R234. 10.1093/hmg/ddi330 16150739

[B52] GribnauJ.LuikenhuisS.HochedlingerK.MonkhorstK.JaenischR. (2005). X chromosome choice occurs independently of asynchronous replication timing. J. Cell Biol. 168, 365–373. 10.1083/jcb.200405117 15668296PMC2171734

[B53] GuoY.XuQ.CanzioD.ShouJ.LiJ.GorkinD. U. (2015). CRISPR Inversion of CTCF sites alters genome topology and enhancer/promoter function. Cell 162, 900–910. 10.1016/j.cell.2015.07.038 26276636PMC4642453

[B54] GuvenG.Erginel-UnaltunaN.SamanciB.GulecC.HanagasiH.BilgicB. (2019). A patient with early-onset Alzheimer's disease with a novel PSEN1 p.Leu424Pro mutation. Neurobiol. Aging. 84, 238.e1–238.e4. 10.1016/j.neurobiolaging.2019.05.014 31296348

[B55] HaackT. B.HogarthP.GregoryA.ProkischH.HayflickS. J. (2013). BPAN: the only X-linked dominant NBIA disorder. Int. Rev. Neurobiol. 110, 85–90. 10.1016/b978-0-12-410502-7.00005-3 24209435

[B56] HardyJ.GoateA.OwenM.RossorM. (1989). Presenile dementia associated with mosaic trisomy 21 in a patient with a Down syndrome child. Lancet 2, 743. 10.1016/s0140-6736(89)90805-2 2570989

[B57] Hauss-WegrzyniakB.DobrzanskiP.StoehrJ. D.WenkG. L. (1998). Chronic neuroinflammation in rats reproduces components of the neurobiology of Alzheimer's disease. Brain Res. 780, 294–303. 10.1016/s0006-8993(97)01215-8 9507169

The article "The X Files: “The Mystery of X Chromosome Instability in Alzheimer’s Disease”" was published in 2020. Journal: Front Genet.

[B58] HongD. S.ReissA. L. (2014). Cognitive and neurological aspects of sex chromosome aneuploidies. Lancet Neurol. 13, 306–318. 10.1016/s1474-4422(13)70302-8 24556008

[B60] IourovI. Y.VorsanovaS. G.YurovY. B. (2006). Chromosomal variation in mammalian neuronal cells: known facts and attractive hypotheses. Int. Rev. Cytol. 249, 143–191. 10.1016/s0074-7696(06)49003-3 16697283

[B61] IourovI. Y.VorsanovaS. G.YurovY. B. (2008). Molecular cytogenetics and cytogenomics of brain diseases. Curr. Genomics 9, 452–465. 10.2174/138920208786241216 19506734PMC2691674

[B59] IourovI. Y.VorsanovaS. G.LiehrT.YurovY. B. (2009). Aneuploidy in the normal, Alzheimer's disease and ataxia-telangiectasia brain: differential expression and pathological meaning. Neurobiol. Dis. 34, 212–220. 10.1016/j.nbd.2009.01.003 19344645

[B62] IourovI. Y.VorsanovaS. G.YurovY. B. (2010). Somatic genome variations in health and disease. Curr. Genomics 11, 387–396. 10.2174/138920210793176065 21358982PMC3018718

[B63] KhalifaO.PersY. M.FerreiraR.SenechalA.JorgensenC.ApparaillyF. (2016). X-Linked miRNAs associated with gender differences in rheumatoid arthritis. Int. J. Mol. Sci. 17, 1852–1863. 10.3390/ijms17111852 PMC513385227834806

[B64] KrsticD.MadhusudanA.DoehnerJ.VogelP.NotterT.ImhofC. (2012). Systemic immune challenges trigger and drive Alzheimer-like neuropathology in mice. J. Neuroinflammation 9, 151. 10.1186/1742-2094-9-151 22747753PMC3483167

[B65] LaskowskiA. I.NeemsD. S.LasterK.Strojny-OkyereC.RiceE. L.KoniecznaI. M. (2019). Varying levels of X chromosome coalescence in female somatic cells alters the balance of X-linked dosage compensation and is implicated in female-dominant systemic lupus erythematosus. Sci. Rep. 9, 8011. 10.1038/s41598-019-44229-9 31142749PMC6541617

[B66] LaumonnierF.CuthbertP. C.GrantS. G. (2007). The role of neuronal complexes in human X-linked brain diseases. Am. J. Hum. Genet. 80, 205–220. 10.1086/511441 17236127PMC1785339

[B67] Le GallJ.NizonM.PichonO.AndrieuxJ.Audebert-BellangerS.BaronS. (2017). Sex chromosome aneuploidies and copy-number variants: a further explanation for neurodevelopmental prognosis variability? Eur. J. Hum. Genet. 25, 930–934. 10.1038/ejhg.2017.93 28612834PMC5567159

[B68] LopesA. M.RossN.CloseJ.DagnallA.AmorimA.CrowT. J. (2006). Inactivation status of PCDH11X: sexual dimorphisms in gene expression levels in brain. Hum. Genet. 119, 267–275. 10.1007/s00439-006-0134-0 16425037

[B69] LuT.AronL.ZulloJ.PanY.KimH.ChenY. (2014). REST and stress resistance in ageing and Alzheimer's disease. Nature 507, 448–454. 10.1038/nature13163 24670762PMC4110979

The article "The X Files: “The Mystery of X Chromosome Instability in Alzheimer’s Disease”" was published in 2020. Journal: Front Genet.

[B70] LuperchioT. R.WongX.ReddyK. L. (2014). Genome regulation at the peripheral zone: lamina associated domains in development and disease. Curr. Opin. Genet. Dev. 25, 50–61. 10.1016/j.gde.2013.11.021 24556270

[B71] LyonM. F. (1961). Gene action in the X-chromosome of the mouse (Mus musculus L.). Nature 190, 372–373. 10.1038/190372a0 13764598

[B72] MadrigalI.Rodríguez-RevengaL.ArmengolL.GonzálezE.RodriguezB.BadenasC. (2007). X-chromosome tiling path array detection of copy number variants in patients with chromosome X-linked mental retardation. BMC Genomics 8, 443. 10.1186/1471-2164-8-443 18047645PMC2234261

[B73] ManzineP. R.PelucchiS.HorstM. A.ValeF. A. C.PavariniS. C. I.AudanoM. (2018). microRNA 221 targets ADAM10 mRNA and is downregulated in Alzheimer's disease. J. Alzheimers Dis. 61, 113–123. 10.3233/jad-170592 29036829

[B74] MaphisN. M.JiangS.BinderJ.WrightC.GopalanB.LambB. T. (2017). Whole Genome Expression Analysis in a Mouse Model of Tauopathy Identifies MECP2 as a Possible Regulator of Tau Pathology. Front. Mol. Neurosci. 10, 69. 10.3389/fnmol.2017.00069 28367114PMC5355442

[B75] MastroeniD.DelvauxE.NolzJ.TanY.GroverA.OddoS. (2015). Aberrant intracellular localization of H3k4me3 demonstrates an early epigenetic phenomenon in Alzheimer's disease. Neurobiol. Aging 36, 3121–3129. 10.1016/j.neurobiolaging.2015.08.017 26553823PMC4838454

[B76] McFarlandK. N.HuizengaM. N.DarnellS. B.SangreyG. R.BerezovskaO.ChaJ. H. (2014). MeCP2: a novel Huntingtin interactor. Hum. Mol. Genet. 23, 1036–1044. 10.1093/hmg/ddt499 24105466PMC3900110

[B77] McGeerP. L.McGeerE. G. (2002). Local neuroinflammation and the progression of Alzheimer's disease. J. Neurovirol. 8, 529–538. 10.1080/13550280290100969 12476347

[B78] MiarA.AlvarezV.CoraoA. I.AlonsoB.DiazM.MenendezM. (2011). Lack of association between protocadherin 11-X/Y (PCDH11X and PCDH11Y) polymorphisms and late onset Alzheimer's disease. Brain Res. 1383, 252–256. 10.1016/j.brainres.2011.01.054 21276771

[B79] MiglioreL.BoniG.BernardiniR.TrippiF.ColognatoR.FontanaI. (2006). Susceptibility to chromosome malsegregation in lymphocytes of women who had a down syndrome child in young age. Neurobiol. Aging 27, 710–716. 10.1016/j.neurobiolaging.2005.03.025 16005550

[B80] MiglioreL.MigheliF.CoppedeF. (2009). Susceptibility to aneuploidy in young mothers of down syndrome children. Sci. World J. 9, 1052–1060. 10.1100/tsw.2009.122 PMC582314519802501

[B81] MinajigiA.FrobergJ. E.WeiC.SunwooH.KesnerB.ColognoriD. (2015). A comprehensive Xist interactome reveals cohesin repulsion and an RNA-directed chromosome conformation. Science 349, aab2276. 10.1126/science.aab2276 PMC484590826089354

The article "The X Files: “The Mystery of X Chromosome Instability in Alzheimer’s Disease”" was published in 2020. Journal: Front Genet.

[B82] MuddashettyR. S.NalavadiV. C.GrossC.YaoX.XingL.LaurO. (2011). Reversible inhibition of PSD-95 mRNA translation by miR-125a, FMRP phosphorylation, and mGluR signaling. Mol. Cell 42, 673–688. 10.1016/j.molcel.2011.05.006 21658607PMC3115785

[B83] MugfordJ. W.StarmerJ.WilliamsR. L.Jr.CalabreseJ. M.MieczkowskiP.YeeD. (2014). Evidence for local regulatory control of escape from imprinted X chromosome inactivation. Genetics 197, 715–723. 10.1534/genetics.114.162800 24653000PMC4063926

[B84] NgK.PullirschD.LeebM.WutzA. (2007). Xist and the order of silencing. EMBO Rep. 8, 34–39. 10.1038/sj.embor.7400871 17203100PMC1796754

[B85] NguyenD. K.DistecheC. M. (2006). Dosage compensation of the active X chromosome in mammals. Nat. Genet. 38, 47–53. 10.1038/ng1705 16341221

[B86] OrstavikK. H. (2009). X chromosome inactivation in clinical practice. Hum. Genet. 126, 363–373. 10.1007/s00439-009-0670-5 19396465

[B87] PeetersS. B.KoreckiA. J.BaldryS. E. L.YangC.TosefskyK.BalatonB. P. (2019). How do genes that escape from X-chromosome inactivation contribute to Turner syndrome? Am. J. Med. Genet. 181, 28–35. 10.1002/ajmg.c.31672 30779428

[B88] PessiaE.MakinoT.Bailly-BechetM.McLysaghtA.MaraisG. A. B. (2012). Mammalian X chromosome inactivation evolved as a dosage-compensation mechanism for dosage-sensitive genes on the X chromosome. Proc. Natl. Acad. Sci. 109, 5346. 10.1073/pnas.1116763109 22392987PMC3325647

[B89] PetersenM. B.KaradimaG.SamaritakiM.AvramopoulosD.VassilopoulosD.MikkelsenM. (2000). Association between presenilin-1 polymorphism and maternal meiosis II errors in down syndrome. Am. J. Med. Genet. 93, 366–372. 10.1002/1096-8628(20000828)93:5<366::AID-AJMG5>3.0.CO;2-G 10951459

[B90] PikeC. J. (2017). Sex and the development of Alzheimer's disease. J. Neurosci. Res. 95, 671–680. 10.1002/jnr.23827 27870425PMC5120614

[B91] PocklingtonA. J.CumiskeyM.ArmstrongJ. D.GrantS. G. (2006). The proteomes of neurotransmitter receptor complexes form modular networks with distributed functionality underlying plasticity and behaviour. Mol. Syst. Biol. 2, 2006 0023. 10.1038/msb4100041 PMC168147416738568

[B92] PomboA.DillonN. (2015). Three-dimensional genome architecture: players and mechanisms. Nat. Rev. Mol. Cell Biol. 16, 245. 10.1038/nrm3965 25757416

[B94] PotterH.GellerL. N. (1996). Alzheimer's disease, Down's syndrome, and chromosome segregation. Lancet 348. 10.1016/s0140-6736(05)64399-1 8691961

[B93] PotterH. (2016). Beyond trisomy 21: phenotypic variability in people with down syndrome explained by further chromosome mis-segregation and mosaic aneuploidy. J. Down Syndr. Chromosom. Abnorm. 2, 1–6. 10.4172/2472-1115.1000109 PMC583706329516054

The article "The X Files: “The Mystery of X Chromosome Instability in Alzheimer’s Disease”" was published in 2020. Journal: Front Genet.

[B95] QuinodozS.GuttmanM. (2014). Long noncoding RNAs: an emerging link between gene regulation and nuclear organization. Trends Cell Biol. 24, 651–663. 10.1016/j.tcb.2014.08.009 25441720PMC4254690

[B96] RaoC. V.FarooquiM.ZhangY.AschA. S.YamadaH. Y. (2018). Spontaneous development of Alzheimer's disease-associated brain pathology in a Shugoshin-1 mouse cohesinopathy model. Aging Cell 17, e12797. 10.1111/acel.12797 29943428PMC6052391

[B97] RaznahanA.ParikshakN. N.ChandranV.BlumenthalJ. D.ClasenL. S.Alexander-BlochA. F. (2018). Sex-chromosome dosage effects on gene expression in humans. Proc. Natl. Acad. Sci. U.S.A. 115, 7398–7403. 10.1073/pnas.1802889115 29946024PMC6048519

[B98] RegenF.Hellmann-RegenJ.CostantiniE.RealeM. (2017). Neuroinflammation and Alzheimer's disease: implications for microglial activation. Curr. Alzheimer Res. 14, 1140–1148. 10.2174/1567205014666170203141717 28164764

[B99] RenaultN. K.DyackS.DobsonM. J.CostaT.LamW. L.GreerW. L. (2007). Heritable skewed X-chromosome inactivation leads to haemophilia a expression in heterozygous females. Eur. J. Hum. Genet. 15, 628–637. 10.1038/sj.ejhg.5201799 17342157

[B100] RenaultN. K.PritchettS. M.HowellR. E.GreerW. L.SapienzaC.OrstavikK. H. (2013). Human X-chromosome inactivation pattern distributions fit a model of genetically influenced choice better than models of completely random choice. Eur. J. Hum. Genet. 21, 1396–1402. 10.1038/ejhg.2013.84 23652377PMC3831084

[B101] SchellenbergG. D.BirdT. D.WijsmanE. M.OrrH. T.AndersonL.NemensE. (1992). Genetic linkage evidence for a familial Alzheimer's disease locus on chromosome 14. Science 258, 668–671. 10.1126/science.1411576 1411576

[B102] SchupfN.KapellD.LeeJ. H.OttmanR.MayeuxR. (1994). Increased risk of Alzheimer's disease in mothers of adults with down's syndrome. Lancet 344, 353–356. 10.1016/s0140-6736(94)91398-6 7914304

[B103] SchupfN.KapellD.NightingaleB.LeeJ. H.MohlenhoffJ.BewleyS. (2001). Specificity of the fivefold increase in AD in mothers of adults with down syndrome. Neurology 57, 979–984. 10.1212/wnl.57.6.979 11571320

[B104] SchurzH.SalieM.TrompG.HoalE. G.KinnearC. J.MöllerM. (2019). The X chromosome and sex-specific effects in infectious disease susceptibility. Hum. Genomics 13, 2. 10.1186/s40246-018-0185-z 30621780PMC6325731

[B105] SelkoeD. J. (2001). Alzheimer's disease results from the cerebral accumulation and cytotoxicity of amyloid beta-protein. J. Alzheimers Dis. 3, 75–80. 10.3233/jad-2001-3111 12214075

[B106] SenA.NelsonT. J.AlkonD. L. (2015). ApoE4 and abeta oligomers reduce BDNF expression *via* HDAC nuclear translocation. J. Neurosci. 35, 7538–7551. 10.1523/jneurosci.0260-15.2015 25972179PMC6705431

The article "The X Files: “The Mystery of X Chromosome Instability in Alzheimer’s Disease”" was published in 2020. Journal: Front Genet.

[B107] SeripaD.PanzaF.FranceschiM.D'OnofrioG.SolfrizziV.DallapiccolaB. (2009). Non-apolipoprotein E and apolipoprotein E genetics of sporadic Alzheimer's disease. Ageing Res. Rev. 8, 214–236. 10.1016/j.arr.2008.12.003 19496238

[B108] ShvetsovaE.SofronovaA.MonajemiR.GagalovaK.DraismaH. H. M.WhiteS. J. (2019). Skewed X-inactivation is common in the general female population. Eur. J. Hum. Genet. 27, 455–465. 10.1038/s41431-018-0291-3 30552425PMC6460563

[B109] SkuseD. H. (2005). X-linked genes and mental functioning. Hum. Mol. Genet. 14 Spec No 1, R27–R32. 10.1093/hmg/ddi112 15809269

[B110] SlooterA. J.de KnijffP.HofmanA.CrutsM.BretelerM. M.Van BroeckhovenC. (1998). Serum apolipoprotein E level is not increased in Alzheimer's disease: the rotterdam study. Neurosci. Lett. 248, 21–24. 10.1016/s0304-3940(98)00339-5 9665654

[B111] SmithM. A. (1998). Alzheimer disease. Int. Rev. Neurobiol. 42, 1–54. 10.1016/s0074-7742(08)60607-8 9476170

[B112] SplinterE.de WitE.NoraE. P.KlousP.van de WerkenH. J.ZhuY. (2011). The inactive X chromosome adopts a unique three-dimensional conformation that is dependent on Xist RNA. Genes Dev. 25, 1371–1383. 10.1101/gad.633311 21690198PMC3134081

[B114] Spremo-PotparevicB.ZivkovicL.DjelicN.BajicV. (2004). Analysis of premature centromere division (PCD) of the X chromosome in Alzheimer patients through the cell cycle. Exp. Gerontol. 39, 849–854. 10.1016/j.exger.2004.01.012 15130680

[B115] Spremo-PotparevicB.ZivkovicL.DjelicN.Plecas-SolarovicB.SmithM. A.BajicV. (2008). Premature centromere division of the X chromosome in neurons in Alzheimer's disease. J. Neurochem. 106, 2218–2223. 10.1111/j.1471-4159.2008.05555.x 18624923PMC2746937

[B113] Spremo-PotparevicB.BajicV.PerryG.ZivkovicL. (2015). Alterations of the X chromosome in lymphocytes of alzheimer's disease patients. Curr. Alzheimer Res. 12, 990–996. 10.2174/1567205012666151027124154 26502819

[B116] SudbrakR.WieczorekG.NuberU. A.MannW.KirchnerR.ErdoganF. (2001). X chromosome-specific cDNA arrays: identification of genes that escape from X-inactivation and other applications. Hum. Mol. Genet. 10, 77–83. 10.1093/hmg/10.1.77 11136717

[B117] SunB. K.LeeJ. T. (2006). “X-Chromosome Inactivation,” in Encyclopedic Reference of Genomics and Proteomics in Molecular Medicine (Berlin, Heidelberg: Springer Berlin Heidelberg), 2013–2019.

[B118] TamG. W.RedonR.CarterN. P.GrantS. G. (2009). The role of DNA copy number variation in schizophrenia. Biol. Psychiatry 66, 1005–1012. 10.1016/j.biopsych.2009.07.027 19748074

[B119] UeberhamU.ArendtT. (2005). The expression of cell cycle proteins in neurons and its relevance for Alzheimer's disease. Curr. Drug Targets CNS Neurol. Disord. 4, 293–306. 10.2174/1568007054038175 15975031

The article "The X Files: “The Mystery of X Chromosome Instability in Alzheimer’s Disease”" was published in 2020. Journal: Front Genet.

[B120] VestR. S.PikeC. J. (2013). Gender, sex steroid hormones, and Alzheimer's disease. Horm. Behav. 63, 301–307. 10.1016/j.yhbeh.2012.04.006 22554955PMC3413783

[B121] VorsanovaS. G.YurovY. B.KolotiiA. D.SolovievI. V. (2001). FISH analysis of replication and transcription of chromosome X loci: new approach for genetic analysis of Rett syndrome. Brain Dev. 23 Suppl 1, S191–S195. 10.1016/s0387-7604(01)00364-3 11738871

[B122] WaniA.GuptaM.AhmadM.ShahA. M.AhsanA. U.QaziP. H. (2019). Alborixin clears amyloid-β by inducing autophagy through PTEN-mediated inhibition of the AKT pathway. Autophagy 15, 1810–1828. 10.1080/15548627.2019.1596476 30894052PMC6735498

[B123] WestraJ. W.RiveraR. R.BushmanD. M.YungY. C.PetersonS. E.BarralS. (2010). Neuronal DNA content variation (DCV) with regional and individual differences in the human brain. J. Comp. Neurol. 518, 3981–4000. 10.1002/cne.22436 20737596PMC2932632

[B124] WilsonN. D.RossL. J. N.CloseJ.MottR.CrowT. J.VolpiE. V. (2007). Replication profile of PCDH11X and PCDH11Y, a gene pair located in the non-pseudoautosomal homologous region Xq21.3/Yp11.2. Chromosome Res. Int. J. Mol. Supramol. Evol. Aspects Chromosome Biol. 15, 485–498. 10.1007/s10577-007-1153-y PMC277938517671842

[B125] Winick-NgW.RylettR. J. (2018). Into the fourth dimension: dysregulation of genome architecture in aging and Alzheimer's disease. Front. Mol. Neurosci. 11, 60. 10.3389/fnmol.2018.00060 29541020PMC5835833

[B126] WisemanF. K.PulfordL. J.BarkusC.LiaoF.PorteliusE.WebbR. (2018). Trisomy of human chromosome 21 enhances amyloid-beta deposition independently of an extra copy of APP. Brain 141, 2457–2474. 10.1093/brain/awy159 29945247PMC6061702

[B127] WuZ. C.YuJ. T.WangN. D.YuN. N.ZhangQ.ChenW. (2010). Lack of association between PCDH11X genetic variation and late-onset Alzheimer's disease in a Han Chinese population. Brain Res. 1357, 152–156. 10.1016/j.brainres.2010.08.008 20707987

[B128] YuanD.XiuJuanW.YanZ.JunQinL.FangX.ShirongY. (2015). Use of X-chromosome inactivation pattern to analyze the clonality of 14 female cases of kaposi sarcoma. Med. Sci. Monitor Basic Res. 21, 116–122. 10.12659/MSMBR.894089 PMC448233226076995

[B129] YudowskiG. A.OlsenO.AdesnikH.MarekK. W.BredtD. S. (2013). Acute inactivation of PSD-95 destabilizes AMPA receptors at hippocampal synapses. PLoS One 8, e53965. 10.1371/journal.pone.0053965 23342049PMC3546964

[B131] YurovY. B.IourovI. Y.VorsanovaS. G.LiehrT.KolotiiA. D.KutsevS. I. (2007). Aneuploidy and confined chromosomal mosaicism in the developing human brain. PLoS One 2, e558. 10.1371/journal.pone.0000558 17593959PMC1891435

[B133] YurovY. B.VorsanovaS. G.LiehrT.KolotiiA. D.IourovI. Y. (2014). X chromosome aneuploidy in the Alzheimer's disease brain. Mol. Cytogenet. 7, 20. 10.1186/1755-8166-7-20 24602248PMC3995993

The article "The X Files: “The Mystery of X Chromosome Instability in Alzheimer’s Disease”" was published in 2020. Journal: Front Genet.

[B132] YurovY. B.VorsanovaS. G.IourovI. Y. (2019). Chromosome instability in the neurodegenerating brain. Front. Genet. 10, 892. 10.3389/fgene.2019.00892 31616475PMC6764389

[B130] YurovY. B. (2017). “FISH-Based Assays for Detecting Genomic (Chromosomal) Mosaicism in Human Brain Cells,” in Genomic Mosaicism in Neurons and Other Cell Types. Eds. FradeJ. M.GageF. (London, UK: Springer Nature).

[B134] ZivkovićL.Spremo-PotparevićB.Plecas-SolarovićB.DjelićN.OcićG.SmiljkovićP. (2010). Premature centromere division of metaphase chromosomes in peripheral blood lymphocytes of Alzheimer's disease patients: relation to gender and age. J. Gerontol. Ser. A Biol. Sci. Med. Sci. 65, 1269–1274. 10.1093/gerona/glq148 20805239PMC2990265

[B135] ZivkovicL.Spremo-PotparevicB.SiedlakS. L.PerryG.Plecas-SolarovicB.MilicevicZ. (2013). DNA damage in Alzheimer disease lymphocytes and its relation to premature centromere division. Neurodegener. Dis. 12, 156–163. 10.1159/000346114 23406622

[B137] ZubenkoG. S.StifflerJ. S.HughesH. B.HurttM. R.KaplanB. B. (1998). Initial results of a genome survey for novel Alzheimer's disease risk genes: association with a locus on the X chromosome. Am. J. Med. Genet. 81, 196–205. 10.1002/(sici)1096-8628(19980207)81:1<98::aid-ajmg17>3.0.co;2-r 9613863

[B136] ZubenkoG. S.HughesH. B.StifflerJ. S. (1999). Clinical and neurobiological correlates of DXS1047 genotype in Alzheimer's disease. Biol. Psychiatry 46, 173–181. 10.1016/s0006-3223(99)00035-9 10418691

